The article "Fibroblast growth factor receptor 1 is principally responsible for fibroblast growth factor 2-induced catabolic activities in human articular chondrocytes" was retracted in 2024. Reason: fabricated or falsified data.

# Fibroblast growth factor receptor 1 is principally responsible for fibroblast growth factor 2-induced catabolic activities in human articular chondrocytes

**DOI:** 10.1186/ar3441

**Published:** 2011-08-11

**Authors:** Dongyao Yan, Di Chen, Simon M Cool, Andre J van Wijnen, Katalin Mikecz, Gillian Murphy, Hee-Jeong Im

**Affiliations:** 1 Department of Biochemistry, Rush University Medical Center, 1735 W Harrison Street, Chicago, IL 60612, USA; 2 Department of Internal Medicine, Section of Rheumatology, Rush University Medical Center, 1735 W Harrison Street, Chicago, IL 60612, USA; 3 Orthopedic Surgery, Rush University Medical Center, 1735 W Harrison Street, Chicago, IL 60612, USA; 4 Department of Bioengineering, University of Illinois, 1304 West Springfield Avenue, Chicago, IL 60612, USA; 5 Department of Stem Cells and Tissue Repair, Institute of Medical Biology, A*STAR, 8A Biomedical Grove, #06-06 Immunos, 138648 Singapore; 6 Division of Musculoskeletal Oncology, Department of Orthopaedic Surgery, Yong Loo Lin School of Medicine, National University of Singapore, 5 Lower Kent Ridge Road, 119074 Singapore; 7 Department of Cell Biology, University of Massachusetts Medical School, 55 Lake Avenue North, Worcester, MA 01655, USA; 8 Department of Oncology, Cambridge University, Cancer Research Institute, Li Ka Shing Center, Robinson Way, Cambridge, CB2 ORE, UK

## Abstract

**Introduction:**

Cartilage degeneration driven by catabolic stimuli is a critical pathophysiological process in osteoarthritis (OA). We have defined fibroblast growth factor 2 (FGF-2) as a degenerative mediator in adult human articular chondrocytes. Biological effects mediated by FGF-2 include inhibition of proteoglycan production, up-regulation of matrix metalloproteinase-13 (MMP-13), and stimulation of other catabolic factors. In this study, we identified the specific receptor responsible for the catabolic functions of FGF-2, and established a pathophysiological connection between the FGF-2 receptor and OA.

**Methods:**

Primary human articular chondrocytes were cultured in monolayer (24 hours) or alginate beads (21 days), and stimulated with FGF-2 or FGF18, in the presence or absence of FGFR1 (FGF receptor 1) inhibitor. Proteoglycan accumulation and chondrocyte proliferation were assessed by dimethylmethylene blue (DMMB) assay and DNA assay, respectively. Expression of FGFRs (FGFR1 to FGFR4) was assessed by flow cytometry, immunoblotting, and quantitative real-time PCR (qPCR). The distinctive roles of FGFR1 and FGFR3 after stimulation with FGF-2 were evaluated using either pharmacological inhibitors or FGFR small interfering RNA (siRNA). Luciferase reporter gene assays were used to quantify the effects of FGF-2 and FGFR1 inhibitor on MMP-13 promoter activity.

**Results:**

Chondrocyte proliferation was significantly enhanced in the presence of FGF-2 stimulation, which was inhibited by the pharmacological inhibitor of FGFR1. Proteoglycan accumulation was reduced by 50% in the presence of FGF-2, and this reduction was successfully rescued by FGFR1 inhibitor. FGFR1 inhibitors also fully reversed the up-regulation of MMP-13 expression and promoter activity stimulated by FGF-2. Blockade of FGFR1 signaling by either chemical inhibitors or siRNA targeting FGFR1 rather than FGFR3 abrogated the up-regulation of matrix metalloproteinases 13 (MMP-13) and a disintegrin and metalloproteinase with a thrombospondin type 1 motif 5 (ADAMTS5), as well as down-regulation of aggrecan after FGF-2 stimulation. Flow cytometry, qPCR and immunoblotting analyses suggested that FGFR1 and FGFR3 were the major FGFR isoforms expressed in human articular chondrocytes. FGFR1 was activated more potently than FGFR3 upon FGF-2 stimulation. In osteoarthritic chondrocytes, FGFR3 was significantly down regulated (*P *< 0.05) with a concomitant increase in the FGFR1 to FGFR3 expression ratio (*P *< 0.05), compared to normal chondrocytes. Our results also demonstrate that FGFR3 was negatively regulated by FGF-2 at the transcriptional level through the FGFR1-ERK (extracellular signal-regulated kinase) signaling pathway in human articular chondrocytes.

**Conclusions:**

FGFR1 is the major mediator with the degenerative potential in the presence of FGF-2 in human adult articular chondrocytes. FGFR1 activation by FGF-2 promotes catabolism and impedes anabolism. Disruption of the balance between FGFR1 and FGFR3 signaling ratio may contribute to the pathophysiology of OA.

## Introduction

Osteoarthritis (OA) is a debilitating disease afflicting millions of people worldwide, which imposes a tremendous burden upon society. OA is a multifactorial heterogeneous disease that is influenced by both genetic and environmental factors [1]. A wide array of enzymes, such as matrix metalloproteinases (MMPs) and a disintegrin and metalloproteinase with a thrombospondin type 1 motif (ADAMTS), and pro-inflammatory cytokines, have been implicated in pathological processes associated with OA, such as cartilage degradation, synovial inflammation and bone abnormalities [2]. Notably, the products of cartilage degeneration not only further promote matrix degradation, but also stimulate the synovium to overproduce inflammatory mediators and degrading proteases, which, in turn, exacerbate cartilage matrix loss [2]. Such autocrine and paracrine loops perpetuate joint destruction, frequently resulting in irreversible disease progression.

Progressive damage to articular cartilage is a hallmark of OA, and a principal cause of tissue break-down is the destruction rather than formation of the cartilage extracellular matrix by chondrocytes. Thus, metabolic homeostasis is perturbed at the cellular level in OA because chondrocyte catabolism predominates over anabolism resulting in net cartilage degeneration. Elevated levels of pro-inflammatory cytokines, inflammatory mediators and certain growth factors potently heighten the expression of matrix-degrading enzymes. Destructive proteases such as MMP-13 and ADAMTS-5 are able to cleave major components in the extracellular matrix of chondrocytes, including type II collagen and aggrecan [3,4]. In response to tissue damage, chondrocytes make attempts at matrix repair, but they often fail to restore the eroded cartilage to its original pristine hyaline state, due to multiple impairing mechanisms [5-8].

FGF-2 participates in the regulation of cartilage homeostasis in addition to its well-established mitogenic role [9]. Released from the extracellular matrix upon tissue injury [10], FGF-2 stimulates MMP-13 expression, which may accelerate cartilage degradation [11]. In both articular chondrocytes and meniscal chondrocytes, FGF-2 alters the ratio between type II and type I collagen, thus possibly resulting in the formation of fibrocartilage, a defective substitute for healthy hyaline cartilage [12,13]. In porcine articular chondrocytes, FGF-2 antagonizes IGF-1/TGF-β-mediated type II collagen and decorin production [14]. Moreover, FGF-2 potently inhibits IGF-1/BMP-7-enhanced proteoglycan accumulation and synthesis in human articular chondrocytes, even though it stimulates proliferation, and markedly affects physical properties of normal cartilage [5,15]. Recent studies by others, suggest a chondroprotective role of FGF-2 in cartilage biology, which merits additional studies to resolve the physiological complexities linked to the opposing biological functions of FGF-2 in human articular cartilage [16,17].

Our group has clearly established that FGF-2 exerts catabolic effects in primary human articular chondrocytes cultured *ex vivo*, thus mechanistically predicting cartilage degradation in human patients. Previously, we showed that FGF-2 inhibits the synergistic anabolic effects of IGF-1 and BMP-7, and also stimulates MMP-13 expression *via *protein kinase C δ (PKCδ)-mediated activation of multiple MAP kinases (ERK1/2, p38 and JNK) [5,18]. We also showed that FGF-2 activates the NFκB pathway, which converges with the MAP kinase pathway on the activation of transcription factor Elk-1 to stimulate MMP-13 transcription [19].

There are four different isoforms of FGF receptors (FGFR1 to FGFR4) that are responsible for the biological impact of FGF-2 through the developmental stages [20]. It is still not clear which receptor(s) mediate the catabolic and/or anti-anabolic signaling by FGF-2 as we previously observed, and what other target genes than MMP-13 are regulated by FGF-2 in human adult articular cartilage [5,18,19]. In this study, we examined which of the main FGFR isoforms mediate the biological effects of FGF-2, characterized critical FGF-2-regulated genes that depend on FGF-2/receptor signaling. We also determined the potential pathological alterations in the expression profiles of FGFR isoforms by comparing cartilage from healthy (Collin' grade 0 or 1) and age- and gender-matched osteoarthritic knee joints (surgically removed).

## Materials and methods

### Materials

Human recombinant FGF-2 was purchased from the National Cancer Institute (Bethesda, MD, USA). Human recombinant FGF18 was purchased from PeproTech (Rocky Hill, NJ, USA). Antibodies against human Flg (FGFR1), Bek (FGFR2), FGFR3, FGFR4, and phospho-Tyrosine (PY99) were purchased from Santa Cruz Biotechnology (Santa Cruz, CA, USA). The antibody against human β-actin was purchased from Abcam (Cambridge, MA, USA). The antibody against human ADAMTS5 was purchased from Millipore (Billerica, MA, USA) and the antibody against MMP-13 and FGFR1 neutralizing antibody were provided by courtesy of Dr. Gillian Murphy and Dr. Simon Cool, respectively. The MMP-13 antibody was described previously [21]. A full characterization of the neutralizing antibody against FGFR1 is provided elsewhere [22]. The titer of the latter antibody is equal or higher than 1:200,000 as determined by standard enzyme-linked immunosorbent assay (ELISA). Pharmacological inhibitor SU5402 (FGFR1i) and PD98059 (ERKi) were purchased from Calbiochem/EMD Chemicals (Gibbstown, NJ, USA). The SU5402 concentrations used in this study (5 μM and 2 μM) did not lead to significant inhibition of FGFR3 phosphorylation, as determined by immunoprecipitation and immunoblotting (data not shown). Stealth small interfering RNA (siRNA) targeting FGFR1 and FGFR3 were purchased from Invitrogen (Carlsbad, CA, USA).

### Chondrocyte isolation and culture

Normal human knee cartilage tissues were obtained within 24 hours of death of donors (age ranging from 40 to 65) from the Gift of Hope Organ and Tissue Donor Network (Elmhurst, IL, USA) with approval by the local ethics committee and consent from the families. Prior to dissection, each specimen was graded for overall degenerative changes based on the modified 5-point scale of Collins [23]. Surgically removed cartilage from OA patients (age ranging from 40 to 65) were obtained from the Orthopedic Tissue and Implant Repository Study with consent from the patients. Human tissues were handled according to the guidelines of the Human Investigation Committee of Rush University Medical Center.

Chondrocytes were isolated by enzymatic digestion of cartilage using Pronase for one hour, followed by overnight digestion with collagenase-P as described previously [5,24]. For monolayer cultures, isolated cells were washed and suspended in culture media at 3 × 10^6 ^cells/mL, and seeded onto 12-well plates using 1 mL media/well. Cells were maintained in Dulbecco's Modified Eagle's Medium (DMEM)/F-12 (1:1) containing 10% fetal bovine serum and antibiotics (complete media) for three days before the treatments. For alginate bead culture, cells were suspended in alginate (2 × 10^6 ^cells/mL) immediately after enzymatic digestion and washing steps, and beads were formed in CaCl_2 _solution, as described previously [25,26]. Beads were cultured in DMEM/F-12 medium (1:1), supplemented with 1% mini-ITS+ premix and 0.1% ascorbic acid, at eight beads per well in 24-well plates. Chondrocytes used for profiling FGFR isoform expression were processed immediately after cell isolation from cartilage.

### Chondrocyte stimulation and immunoblotting

Prior to treatments, chondrocytes were growth factor deprived in serum-free DMEM/F-12 (1:1) for 24 hours. Media were replaced again with fresh serum-free DMEM/F-12 (1:1) two hours before stimulation. When inhibitors were applied, cells were pre-incubated with individual pathway-specific inhibitors for one hour before stimulation with FGF-2 (100 ng/mL). After terminating the experiments, conditioned media and whole cell lysates were collected. Media were stored at 4°C with 0.1% NaN_3_, and used within five days. Cell lysates were prepared using modified cell lysis RIPA buffer: 20 mM Tris (pH 7.5), 150 mM NaCl, 1 mM EDTA, 1 mM EGTA, 1% Nonidet P-40, 0.25% deoxycholate, 2.5 mM sodium pyrophosphate, 1 mM glycerol phosphate, 1 mM NaVO_4_, and 2 mM phenylmethylsulfonyl fluoride (Sigma, St Louis, MO, USA). Total protein concentrations of the cell lysates were determined using the bicinchoninic acid (BCA) assay (Thermo Scientific, Rockford, IL, USA). Equal amounts of protein were resolved in 10% SDS-polyacrylamide gels and transferred to nitrocellulose membrane for immunoblotting analyses as described previously [24]. Immunoreactivity was visualized using an ECL system (Pierce, Rockford, IL, USA).

### Immunoprecipitation

Whole cell lysates were prepared as described above and centrifuged at 12,500 rpm for 20 minutes. Supernatants were transferred and incubated with antibody against FGFR1 or FGFR3 immobilized to Protein A agarose beads (Thermo Scientific, Rockford, IL, USA). Beads were maintained in homogenous suspension overnight at 4°C using a rotary wheel that supports 'end-over-end' mixing. Beads were then washed three times with binding buffer (0.14 M NaCl, 0.008 M sodium phosphate, 0.002 M potassium phosphate, 0.01 M KCl, pH 7.4). The samples were eluted and subjected to SDS-PAGE.

### Total RNA extraction, cDNA synthesis, and quantitative real-time PCR

Total RNA from normal and osteoarthritic human articular chondrocytes was isolated using Trizol reagent (Invitrogen, Carlsbad, CA, USA) following the instructions provided by the manufacturer. Reverse transcription (RT) was carried out with 1 μg total RNA using ThermoScript ^TM ^RT-PCR system (Invitrogen) for first strand cDNA synthesis. For real-time PCR, cDNA was amplified using MyiQ Real-Time PCR Detection System (Bio-Rad, Hercules, CA, USA). Relative gene expression was determined using the ^ΔΔ^C_T _method, using detailed guidelines provided by the manufacturer (Bio-Rad). 18S rRNA and GAPDH were used as internal controls for normalization. The standard deviations in samples were calculated using data from at least five different donors in independent experiments. The primer sequences are summarized in Table 1.

**Table 1:** Real-time PCR primer sequences

Gene	Primer Sequence (5'→3')	NCBI Gene Number	Anneal T_m_
MMP13	F: ACCCTGGAGCACTCATGTTTCCTA R: TGGCATCAAGGGATAAGGAAGGGT	NM_002427.3	60°C
ADAMTS5	F: CTGTGACGGCATCATTGGCTCAAA R: TTCAGGAATCCTCACCACGTCAGT	NM_007038.3	60°C
ACAN	F: TCTTGGAGAAGGGAGTCCAACTCT R: ACAGCTGCAGTGATGACCCTCAGA	NM_001135.3	60°C
FGFR1	F: AACCTGACCACAGAATTGGAGGCT R: ATGCTGCCGTACTCATTCTCCACA	NM_023110.2	60°C
FGFR2	F: TGATGGACTTCCTTATGTCCGCGT R: AGCGTCCTCTTCTGTGACATTGGT	NM_000141.4	60°C
FGFR3	F: ACCAATGTGTCTTTCGAGGATGCG R: AGAGCACGCAGCTTGTCACATAGA	NM_000142.4	60°C
FGFR4	F: ATGGAACTGGTGTGCTCAAGAAGC R: TTCACATGTCCTCCGACCAACACA	NM_002011.3	60°C
18S rRNA	F: CGGCTACCACATCCAAGGAA R: GCTGGAATTACCGCGGCT	NR_003286.2	60°C
GAPDH	F: TCGACAGTCAGCCGCATCTTCTTT R: GCCCAATACGACCAAATCCGTTGA	NM_002046.3	60°C

ACAN, aggrecan core protein; ADAMTS5, a disintegrin and metalloproteinase with a thrombospondin type 1 motif 5; FGFR, fibroblast growth factor receptor; GAPDH, glyceraldehyde 3-phosphate dehydrogenase; MMP13, matrix metalloproteinase-13.

### Dimethylmethylene blue (DMMB) assay and DNA assay

Cultured cells on alginate beads were collected and processed for quantitative assays using the DMMB binding method, as previously described [26,27]. The pH of DMMB solution used in this study was 1.5, in order to minimize the interfering effect of alginate, as previously demonstrated [28]. The proteoglycan levels in the cell-associated matrix were measured. Cell viability and cell numbers were determined using PicoGreen (Invitrogen), as previously described [26].

### Transient transfection

Nucleofection was optimized for human articular chondrocytes based on the manual of the Nucleofector^™ ^kit (Lonza, Walkersville, MD, USA) as described previously [29,30]. Chondrocytes were cultivated for three days before transfection. For FGFR knockdown experiments, siRNA at a concentration of 200 nM (20 pmol/sample) was used during transfection. After 48 hours, cell lysates were subjected to SDS-PAGE and immunoblotting for validation of successful knockdown. In parallel, stimulations were performed 48 hours after the transfection. In promoter activity assays, as internal control for transfection efficiency, the *Renilla *Luciferase vector (pRL-TK) was co-transfected with the MMP-13 promoter/firefly luciferase constructs as we described previously [18]. Both *Renilla *and firefly luciferase activity were measured simultaneously using a dual-luciferase reporter assay system (Promega, Madison, WI, USA) and a luminometer (Berthold, Huntsville, AL, USA).

### Flow cytometry analysis

Immunofluorescence labeling of FGFRs was performed as previously described [31]. Human articular chondrocytes were incubated with anti-CD32/CD16 monoclonal antibody to block Fc receptor-mediated nonspecific antibody binding. Primary antibodies against FGFR1, FGFR2, FGFR3, and FGFR4 were incubated with cells, followed by addition of secondary antibody, goat-anti-rabbit Alexa Fluor 488 (Invitrogen). Cells were also incubated with goat-anti-rabbit Alexa Fluor 488, or non-immune rabbit serum plus goat-anti-rabbit Alexa Fluor 488 as controls. FGFRs present on the plasma membrane of chondrocytes were analyzed using a FACS Calibur instrument and CellQuest software (BD Flow Cytometry Systems, San Jose, CA, USA).

### Statistical analysis

Statistical significance was determined by Student's *t*-test, or one-way repeated measures ANOVA followed by Sidak *post-hoc *test using the SPSS 17 program. *P*-values lower than 0.05 were considered to be statistically significant in each test.

## Results

### FGF-2-mediated cellular proliferation and proteoglycan loss is *via *FGFR1 in human articular chondrocytes

Previously, we reported FGF-2-mediated cell proliferation and significant proteoglycan loss in human articular cartilage using *in vitro *and *ex vivo *explant culture systems [5]. Dynamic interactions of FGF-2 with its cognate receptors, FGFR1 and FGFR3 were shown to elicit distinctive biological responses. FGF-2 binds to all FGFR isoforms, yet with higher affinity to FGFR1 and FGFR3 [32]. We investigated which specific FGFR isoforms are responsible for the FGF-2-mediated cellular proliferation and proteoglycan loss.

Human articular chondrocytes in alginate beads were incubated with FGF-2 for 21 days in the presence or absence of a pharmacological inhibitor that blocks the tyrosine kinase activity of FGFR1 (SU5402, 2 μM) or a neutralizing antibody directed against FGFR1 antibody [22]. Treatment with FGF18 was included in parallel, because its pro-anabolic activity for matrix formation is exclusively mediated through activation of FGFR3 in human articular cartilage [33]. Accumulated cell-associated proteoglycan and cellular proliferation were assessed by DMMB assay. Our results show that FGF-2 significantly reduced proteoglycan production, whereas FGF18 was pro-anabolic (Figure 1A), consistent with previous findings [5,33,34]. In parallel, we found that FGF-2 but not FGF18 significantly induced cell proliferation (up to two-fold) (Figure 1B). This reduction of proteoglycan biosynthesis and stimulation of proliferation by FGF-2 were each completely abolished by co-incubation with either the pharmacological inhibitor of FGFR1 (2 μM) or the neutralizing anti-FGFR1 antibody, while neither agent affected FGF18-mediated proteoglycan production (Figure 1A, B). Consistent with our previous report, FGF-2 did not alter cell survival, suggesting FGF-2 does not impact cell death (data not shown) [5]. These data indicate that the biological impact of FGF-2 is achieved *via *the activation of FGFR1 but not FGFR3. Our data corroborate the current concept that FGFR1 and FGFR3 have distinct biological roles in articular chondrocytes, and that activation of FGFR3 by FGF18 is anabolic for human articular cartilage homeostasis [33,34].

**Figure 1:** **The effect of FGF-2 on proteoglycan accumulation and cell proliferation**. Human articular chondrocytes were cultured in alginate beads with indicated treatments for 21 days before assaying for proteoglycan and DNA content. **(A) **Proteoglycan accumulation was assessed by dimethylmethylene blue (DMMB) assay, normalized by DNA content. **(B) **Cellular proliferation was quantified by total DNA content in beads from each treatment group. * *P *< 0.05; ** *P *< 0.01. FGF, fibroblast growth factor.

### FGFR1 is responsible for the up-regulation of MMP-13 and ADAMTS5, as well as down-regulation of aggrecan by FGF-2 in human articular chondrocytes

We examined whether FGFR1 is the major receptor responsible for FGF-2-dependent regulation of genes encoding cartilage-degrading enzymes (for example, MMP-13 and ADAMTS5), or major cartilage-related proteoglycans (for example, aggrecan). Because we were interested in investigating the FGFR1-altered transcriptional regulation of the target gene that requires 24-hour incubation, we utilized a monolayer culture system instead of a long-term alginate bead culture system. Human chondrocytes in monolayer were pre-incubated with either SU5402 (5 µM), a pharmacological inhibitor that blocks the tyrosine kinase activity of FGFR1, or a neutralizing antibody directed against FGFR1 (*lane 3 and 4*) followed by stimulation with FGF-2 (100 ng/mL) for 24 hours. Based on a previous report, the SU5402 inhibitor has an IC_50 _of 10 to 20 μM for FGFR1 inhibition [35]. Our empirically determined SU5402 concentration (5 μM) differs from the reported IC_50_, which may be attributed to differences in biological context, experimental conditions and readouts. Conditioned media were collected for analyses of MMP-13 and ADAMTS5 mRNA levels using RT-qPCR with human-specific primer sets for MMP13 and ADAMTS5 that had been validated in our laboratory [36]. Stimulation of cells with FGF-2 alone significantly induced MMP-13 (Figure 2A; *P *< 0.05) and ADAMTS5 (Figure 2B; *P *< 0.05) at both mRNA and protein levels. The biological modulations of FGF-2 on MMP13 and ADAMTS5 were abolished in the presence of either the FGFR1 inhibitor (*P *< 0.05) or the FGFR1 neutralizing antibody (*P *< 0.05). By clear contrast, FGF18 (100 ng/mL), which specifically activates FGFR3, failed to stimulate catabolic enzyme production, and its action was not altered by SU5402 or the neutralizing FGFR1 antibody (data not shown).

**Figure 2:** **Effects mediated by FGFR1 upon FGF-2 binding**. **(A, B, E) **Human articular chondrocytes in monolayer were treated with FGF-2 (100 ng/mL), in the absence or presence of FGFR1 neutralization antibody (1:1,000, 1:200) or SU5402 (5 μM), for 24 hours. In parallel, chondrocytes were transfected with siRNA targeting FGFR1 or FGFR3, and subjected to 24-hour FGF-2 (100 ng/mL) stimulation. Conditioned media were collected for immunoblotting analyses of matrix metalloproteinase-13 (MMP-13) and a disintegrin and metalloproteinase with a thrombospondin type 1 motif 5 (ADAMTS5). Total RNA was extracted for cDNA synthesis and qPCR quantification of gene expression. * *P *< 0.05. **(C) **Chondrocyte lysates were prepared 48 hours after siRNA transfection. The samples were resolved by SDS-PAGE, and immunoblotted for FGFR1 and FGFR3 protein expression. GAPDH was used as a loading control. **(D) **-1600MMP-13 Luciferase-promoter construct was transiently transfected into human articular chondrocytes. The transfected cells were pre-incubated with neutralizing antibody (1:1,000, 1:200) or 5 μM SU5402 for 1 hour, and then stimulated with FGF-2 (100 ng/mL) for 24 hours. The luciferase activity representing MMP-13 promoter activity was measured. A Renilla vector was co-transfected as an internal control for normalization. * *P *< 0.05. ADAMTS, a disintegrin and metalloproteinase with a thrombospondin type 1 motif; FGF, fibroblast growth factor; FGFR, FGF receptor; GAPDH, glyceraldehyde 3-phosphate dehydrogenase; MMP, matrix metalloproteinase; qPCR, quantative polymerase chain reaction; siRNA, small interfering RNA.

To substantiate our findings, human articular chondrocytes in monolayer were transfected with either FGFR1-specific or FGFR3-specific siRNA. Cells were then stimulated with FGF-2 (100 ng/mL), followed by immunoblotting and qPCR to assess MMP-13 and ADAMTS5 expression. Our results indicate that both FGFR1 and FGFR3 were significantly knocked down on their protein levels (Figure 2C). We did not observe any off-target effects of these siRNA on the other FGFR isoforms (data not shown). Consistent with the results acquired using FGFR inhibitors, FGFR1 knockdown resulted in reversal of FGF-2-mediated up-regulation of MMP-13 and ADAMTS5 (Figure 2A, B; *P *< 0.05). By stark contrast, FGFR3 knockdown did not significantly modulate FGF-2-mediated MMP-13 or ADAMTS5 induction (Figure 2A, B), suggesting FGFR1 is the FGFR isoform responsible for the catabolic actions of FGF-2 in articular chondrocytes.

Coherent results were obtained in transient transfection studies that monitored integration of upstream metabolic signals on the promoter of the MMP13 gene. In previous studies, we showed that the first 1.6 kb of the MMP-13 promoter (-1600 MMP-13 Luc reporter construct) responded to FGF-2 stimulation by increasing MMP-13 gene transcription [18]. Here we found that FGF-2-induction of MMP-13 promoter-driven luciferase activity was completely inhibited by SU5402 or neutralizing FGFR1 antibody, with luciferase activity levels returning to the control level (no treatment) (Figure 2D). These results further support our hypothesis that FGFR1 is responsible for the FGF-2-induced MMP-13 expression in human articular chondrocytes.

Administration of FGF-2 significantly reduced the expression of aggrecan (Figure 2E; *P *< 0.05), a major component of proteoglycan in human articular chondrocytes. The inhibition of aggrecan expression by FGF-2 was completely reversed in the presence of either SU5402 (5 µM), or neutralizing FGFR1 antibody in a dose-dependent manner. Likewise, FGFR1 knockdown abolished aggrecan down-regulation by FGF-2, whereas FGFR3 knockdown failed to exert such an effect (Figure 2E; *P *< 0.05). Taken together, our results suggest that pro-catabolic and anti-anabolic biological signals mediated by FGF-2 are relayed through FGFR1 but not FGFR3 in human adult articular chondrocytes.

### FGFR1 and FGFR3 are predominantly expressed in normal human adult articular chondrocytes

We examined the basal expression levels of FGFR family members (FGFR1-4) at the cell surface to understand which receptors mechanistically influence the biological response to FGF-2 in human adult articular cartilage. To determine expression levels of FGFRs, normal knee chondrocytes (Collin's grade 0 or 1, age group from 40 to 65) were subjected to flow cytometric analyses, using anti-FGFR1 to four antibodies. Our results indicate that FGFR3 and FGFR1 were the two most prominent receptors at the cell surface of normal human articular chondrocytes (*n = *3) (Figure 3A). Similarly, cellular mRNA and protein levels of FGFR3 and FGFR1 were predominantly higher than the levels of FGFR2 and FGFR4 based on RT-qPCR data (Figure 3B) and immunoblotting analyses (Figure 3C). Compared with healthy chondrocytes, osteoarthritic chondrocytes did not up-regulate FGFR2 or FGFR4 expression level (data not shown). We also performed FGFR isoform expression analyses using mRNA and protein acquired *via *different procedures (that is, direct extraction from cartilage explants, extraction from cells immediately after enzymatic digestion, and extraction from cells after up to five-day culture), and we did not observe notable differences between these methods regarding FGFR expression levels (data not shown). These results collectively suggest that FGFR3 and FGFR1 are the principal sensors of FGF ligands in articular chondrocytes.

**Figure 3:** **Abundant FGFR1 and FGFR3 expression in articular chondrocytes**. **(A) **Human articular chondrocytes were incubated with anti-CD32/CD16 monoclonal antibody to block nonspecific antibody binding. FGFR1, FGFR2, FGFR3, and FGFR4 antibodies were incubated with cells, followed by incubation with a secondary antibody, goat-anti-rabbit Alexa Fluor 488. Cells were also incubated with goat-anti-rabbit Alexa 488, or non-immune rabbit serum plus goat-anti-rabbit Alexa Fluor 488 as controls. FGFRs on the plasma membrane of chondrocytes were analyzed with a FACS Calibur instrument and CellQuest software. **(B) **Human articular chondrocytes in monolayer were subjected to RNA extraction, cDNA synthesis, and qPCR quantification of FGFR isoform expression. * *P *< 0.05. **(C) **Human articular chondrocytes in monolayer were directly lysed. Equal amounts of total protein were resolved on a SDS-PAGE gel, followed by transfer and immunoblotting of FGFR isoforms. FGF, fibroblast growth factor; FGFR, FGF receptor; qPCR, quantative polymerase chain reaction.

### FGF-2 preferentially activates FGFR1, and to a lesser extent, FGFR3 in human articular chondrocytes

FGF-2 signaling is initiated by ligand binding and subsequent activation of specific FGFRs. Because we observed that FGFR1 and FGFR3 were predominantly expressed in articular chondrocytes, we next asked a question: Which type of FGFR(s) is activated in response to FGF-2? We included FGF18 treatments in the experiments, in parallel for comparison, as FGF18 exclusively activates FGFR3, in human adult articular chondrocytes.

Either FGF-2 or FGF18 (100 ng/mL) was administered in serum-free media to human knee articular chondrocytes in monolayer. Immunoprecipitation (IP) analyses were performed using either FGFR1 or FGFR3 antibody, followed by immunoblotting with a phospho-Tyr (PY99) antibody. In our initial time-course studies, we observed the strongest receptor activation reflected by increased phospho-tyrosine levels within 5 minutes, followed by a rapid decrease within 30 minutes after treatment with FGF-2 or FGF18 (data not shown). Therefore, we selected the five-minute time point to determine specific FGFR activation in response to FGF-2. Our IP results suggest that FGF-2 activated both FGFR1 and FGFR3 with a modest preference towards FGFR1 over FGFR3 in knee articular chondrocytes (Figure 4A). However, FGF18 exclusively activated FGFR3 without detectable activation of FGFR1 (Figure 4B). These results suggest that selective FGFR-ligand interactions drive distinctive signaling pathways and result in differential biological outcomes in human adult articular chondrocytes.

**Figure 4:** **Activation of FGFR1 and FGFR3 by FGF-2**. **(A) **Human articular chondrocytes in monolayer were stimulated with FGF-2 (100 ng/mL) for five minutes before whole cell lysates were prepared. The lysates were incubated with antibody against FGFR1 or FGFR3 in separate tubes. Equal amounts of total protein after immunoprecipitation (IP) were resolved on SDS-PAGE gel, followed by immunoblotting of phospho-tyrosine. Antibody against total FGFR1 or FGFR3 was used to evaluate loading precision. **(B) **Human articular chondrocytes in monolayer were stimulated with FGF18 (100 ng/mL) for five minutes before whole cell lysates were prepared. The following steps were performed as described above. FGF, fibroblast growth factor; FGFR, FGF receptor.

### FGFR3 is down-regulated in OA cells, and is regulated by growth factors

FGFR3 has been shown to elicit anabolic responses in cartilage (for example, FGF18), and *Fgfr3*-knockout mice exhibit premature cartilage degradation and arthritis [34,37]. Previously, we reported hyper-sensitization of osteoarthritic cells to FGF-2 compared to normal chondrocytes [18]. We postulated that the functional differences in the FGF-2 response that are evident between normal and OA cells, or between knee and ankle (unpublished data) is related to altered levels of FGFR subtypes in osteoarthritic chondrocytes. We investigated this hypothesis by comparing FGFR1 and FGFR3 expression at both mRNA and protein levels in normal and osteoarthritic chondrocytes. To minimize biological variability in each group, the specimens were carefully matched for age and gender. Results from RT-qPCR and immunoblot analyses reveal a significant down-regulation of FGFR3 in osteoarthritic cells at both mRNA (Figure 5A; *P *< 0.05) and protein levels (Figure 5B) when compared to normal cells. To understand changes in the relative abundance of FGFR1 and FGFR3 in normal and osteoarthritic specimens, we simultaneously quantified the mRNA levels of FGFR1 and FGFR3 in each donor, and calculated the expression ratios of FGFR1 to FGFR3. The data show that expression ratio of FGFR1 to FGFR3 was significantly increased in OA compared to normal chondrocytes (*P *< 0.05) (Figure 5C). In addition, no apparent correlation between donor age and FGFR expression level was observed (data not shown). Thus, imbalanced FGFR signaling may account for the altered cellular responses to FGF-2 and FGF18 in the osteoarthritic state.

**Figure 5:** **FGFR expression profiles and FGFR3 regulation in articular chondrocytes**. **(A) **Age-matched, normal and osteoarthritic human articular chondrocytes in monolayer were subjected to RNA extraction, cDNA synthesis, and qPCR quantification of FGFR3 expression. **(B) **Age-matched, normal and osteoarthritic human articular chondrocytes were directly lysed for immunoblotting analyses of FGFR3. **(C) **Age-matched, normal and osteoarthritic chondrocytes were subjected to RNA extraction, cDNA synthesis, and qPCR quantification of FGFR1 and FGFR3 expression. The FGFR1 to FGFR3 expression ratio was calculated in each donor. **(D) **Human articular chondrocytes in monolayer were pre-incubated with SU5402 (5 μM) or PD98059 (ERK inhibitor, 50 μM) for 1 hour, and then treated with FGF-2 (100 ng/mL) for 24 hours. In parallel, chondrocytes were transfected with siRNA targeting FGFR1 or FGFR3, and then stimulated by FGF-2 (100 ng/mL) for 24 hours. Total RNA was extracted afterwards for cDNA synthesis and qPCR analyses of FGFR3 expression. * *P *< 0.05. **(E) **Human articular chondrocytes in monolayer were administered with BMP7 (100 ng/mL) and cultured for 24 hours. Total RNA was extracted afterwards for cDNA synthesis and qPCR analyses of FGFR1 and FGFR3 expression. ERK, extracellular signal-regulated kinase; FGF, fibroblast growth factor; FGFR, FGF receptor; qPCR, quantative polymerase chain reaction.

Because progression of OA depends on external signaling ligands (for example, FGFs and BMPs), we investigated whether FGFR3 expression is down-regulated by such factors in chondrocytes. Importantly, administration of FGF-2 significantly decreased the expression level of FGFR3 (Figure 5D; *P *< 0.05). By contrast, BMP-7, a well-known anabolic growth factor in cartilage, markedly increased expression of FGFR3 (Figure 5E; *P *< 0.001) whereas the level of FGFR1 was not significantly modulated in the presence of BMP-7 in human articular chondrocytes. The suppression of FGFR3 expression by FGF-2 was completely abolished in the presence of either FGFR1 inhibitor or FGFR1 neutralizing antibody. Similarly, knockdown of FGFR1 by siRNA rescued FGFR3 suppression in the presence of FGF-2 (Figure 5D; *P *< 0.05). Furthermore, the inhibitor of the ERK MAPK pathway significantly reversed FGF-2-mediated reduction of FGFR3, suggesting that FGF-2-suppression of FGFR3 is *via *FGFR1-ERK/MAPK axis in human articular chondrocytes (Figure 5D).

## Discussion

The balance between FGFR1 and FGFR3 signaling, and the cognate ligands FGF-2 and FGF18, appears to be vital for normal cartilage homeostasis [9]. While FGF-2 binds to all FGFR isoforms *in vitro*, it has greater affinity for FGFR1 and FGFR3 [32]. The anabolic growth factor FGF18 appears to act selectively through FGFR3 to activate distinct downstream pathways in human articular chondrocytes. Of the four receptors for FGFs, we found that FGFR1 and FGFR3 were predominantly expressed in human adult articular chondrocytes. To assess the specific roles of FGFR1 *versus *FGFR3, we used several different experimental criteria. We applied multiple approaches: two inhibitors with distinct modes of action (that is, a chemical inhibitor that blocks the tyrosine kinase activity of FGFR1 and an antibody directed against FGFR1), specific siRNAs that target FGFR1 or FGFR3, as well as comparisons between FGF-2 versus FGF-18 treatments. Published data and our own empirical findings indicate that the chemical inhibitor, the antibody, and the siRNA for FGFR1 each selectively target FGFR1, while FGF-2 and FGF-18 have different downstream effects. These criteria together permit interpretations that the primary functions of FGFR1 and FGFR3 signaling by FGF-2 are distinctive in human adult articular chondrocytes. While contributing functions of FGFR3 in mediating FGF-2 signaling cannot be ruled out categorically, our biological results favor the interpretation that sustained FGF-2/FGFR1 signaling, but not FGFR3 signaling, is primarily responsible for proliferation, pro-catabolism as well as anti-anabolism in adult human articular chondrocytes.

Absence of signaling from FGFR3 was demonstrated to result in increased MMP-13 expression and cartilage degradation, which resembles the osteoarthritic features observed in mice overexpressing MMP-13 [37,38]. This increase in MMP-13 may be due to elevated FGF-2 signaling through FGFR1, which is a dominant, major FGFR subtype in the absence of FGFR3 [33]. The orchestrated and fine-tuned activities of FGFR1 and FGFR3 seem to be essential to extracellular matrix turnover under normal condition [39]. The results presented in this study collectively suggest that FGFR1 and FGFR3 promote catabolism and anabolism, respectively.

Arthritic tissues from OA patients exhibited substantially decreased expression of FGFR3, thus possibly intensifying FGFR1 signaling in human primary knee joint articular chondrocytes. We also found that FGF-2/FGFR1 signaling down-regulated FGFR3 expression in articular chondrocytes. The observation that FGF-2 levels are abnormally elevated in synovial fluid of OA patients fits a molecular model [18], in which FGF-2 initiates a self-reinforcing feedback loop that perpetuates the characteristic degeneration of cartilage in OA, *via *promoting FGF-2/FGFR1 signaling and simultaneously, suppressing FGFR3-related pathways (for example, FGFR3/FGF18 signaling). We observed distinct cellular responses to FGF-2 in different biological contexts (for example, between knee and ankle; normal and OA; young and old, and so on). For example, we consistently observed a more adverse effect of FGF-2 in aged tissue donors ( > 45 years old) with damaged femoral regions (Collin's grade > 2) or clinical OA as previously published [19]. Nevertheless, we do not always observe the same biological effects by FGF-2 using donor tissues from young and normal knee cartilage with Collin's grade 0 or ankle tissues. In particular, although our IP results suggest that FGF-2 more potently activates FGFR1 than FGFR3 in knee articular chondrocytes, we observed differential activities of FGFR1 and FGFR3 in ankle chondrocytes after FGF-2 stimulation, in which FGF-2-induced activation of FGFR3 was as potent as FGFR1 (data not shown). We found these results very interesting as it may provide a molecular mechanistic understanding explaining, in part, why knee joints are more vulnerable to OA compared with ankles. Our data remain more consistent with the initial publications that FGF-2 stimulates catabolism and/or anti-anabolism by inducing cartilage degrading enzymes (for example, MMP1, MMP13) and proteoglycan loss in articular cartilage *in vitro *and *ex vivo *[11,18,19]. However, we are aware of some animal studies that demonstrated that FGF-2-mediates anabolism in knee joints [40]. Although these apparent discrepancies in biological effects are not clearly understood yet, it may result from: age- and grade-dependent differences (correlates with degree of damage) between animal (young and healthy grade 0) and human tissues ( > 45 years old, grade 0/1) or perhaps, disease stage-specific expression/activation pattern of FGF receptors (for example, FGFR1 *versus *FGFR3) as we have shown in this study.

The findings presented here indicate that FGF-2 signaling *via *FGFR1 is required for expression and/or transcriptional regulation of the collagenase MMP-13 and aggrecanase ADAMTS5, as well as suppression of the key anabolic gene aggrecan. Cartilage degradation is linked to ADAMTS5, and specific inhibition of ADAMTS5 is chondroprotective for articular joints [41,42]. Interestingly, we did not observe a significant induction of ADAMTS4 upon FGF-2 stimulation. This finding suggests that ADAMTS5 is preferentially modulated by FGF-2 and may have a selective patho-physiological function that complements MMP-13 and other proteolytic enzymes in OA. Aggrecan turnover occurs in healthy cartilage, and the imbalance between its production and degradation results in defective extracellular matrix [39]. The repression of aggrecan by FGF-2-FGFR1 possibly disrupts normal extracellular matrix metabolism and facilitates further pathogenic progression.

The activation of chondrocyte proliferation by FGF-2/FGFR1 activation observed in this study is consistent with studies in various cell types, including chondrocytic cells [43]. The effect of FGF-2 on stimulating chondrocyte proliferation and proteoglycan-degrading enzymes, and reducing proteoglycan production, may compromise the integrity of the extracellular matrix surrounding newly divided chondrocytes. We previously reported that the endogenous level of FGF-2 is highly increased in osteoarthritic synovial fluids [18]. Increased chondrocyte proliferation was also observed in certain osteoarthritic populations [44]. Therefore, pathologically elevated levels of FGF-2 in osteoarthritic synovial fluid may influence not only cartilage but also the "whole joint organ", including synovial lining and subchondral bone, which may promote fibroblastic proliferation of chondrocytes, resulting in the formation of fibrocartilage with altered biological and biomechanical properties. In addition, neural ingrowth and angiogenesis in synovium, which have been shown in the OA animal model and patients with painful knee joint OA, may be directly and/or indirectly promoted by FGF-2 [45].

Previously, we have shown that FGF-2 potently abrogated BMP-7-mediated proteoglycan synthesis and accumulation [5,46]. Our current study demonstrates that administration of FGF-2 suppressed the FGFR3 gene *via *the activation of ERK/MAPK in human articular chondrocytes. Interestingly, we found that BMP-7 markedly up-regulated FGFR3 expression, and this induction was effectively blocked by the FGF-2-ERK/MAPK axis (unpublished data). It is possible that BMP-7 augments its anabolic activity, in part, *via *induction of FGFR3, thus indirectly potentiating endogenous FGF18-FGFR3 signaling. This may explain the additive effect (if not synergistic) of BMP-7 plus FGF18 on proteoglycan production observed in another set of our studies in human articular chondrocytes (unpublished data). One plausible mechanism is that FGF-2 overrides stimulatory effects of BMP-7 on FGFR3 expression, which negates the responsiveness to FGF18 and diminishes proteoglycan production. These speculations need to be confirmed by a set of experiments in future studies.

## Conclusions

In conclusion, we have provided evidence that FGFR1 primarily transmits detrimental signals in adult human articular chondrocytes upon FGF-2 stimulation, as opposed to FGFR3. FGFR1 signaling leads to inhibition of proteoglycan accumulation, increased catabolic gene expression, and decreased anabolic gene expression. FGFR1 and FGFR3, which represent receptors with the highest affinity for FGF-2, are dominantly expressed in articular chondrocytes. FGFR1 is preferentially activated by FGF-2 over FGFR3, which corroborates the catabolic role of FGF-2. FGFR3 is significantly down regulated in osteoarthritic chondrocytes, and the FGFR1 to FGFR3 expression ratio is elevated in OA. In addition, FGFR3 is down-regulated by FGF-2 signaling through FGFR1-ERK axis. Our findings suggest that FGFR1 specifically has a predominant function in FGF-2-promoted cartilage degeneration and OA pathophysiology.

## Abbreviations

ADAMTS: a disintegrin and metalloproteinase with a thrombospondin type 1 motif; BCA: bicinchoninic acid; DMEM: Dulbecco's modified Eagle's medium; DMMB: dimethylmethylene blue; ERK: extracellular signal-regulated kinase; FGF-2: fibroblast growth factor 2; FGFR: FGF receptor; IP: immunoprecipitation; MMP: matrix metalloproteinase; OA: osteoarthritis; qPCR: quantitative real-time polymerase chain reaction; RT: reverse transcription; siRNA: small interfering RNA.

## Competing interests

The authors declare that they have no competing interests.

## Authors' contributions

DY designed the experiments for this study, acquired the data, interpreted the data, carried out the flow cytometry analysis and drafted the manuscript. DC and H-JI designed the experiments for this study, interpreted the data and drafted the manuscript. SC and GM interpreted the data. KM interpreted the data and carried out the flow cytometry analysis. AW interpreted the data and drafted the manuscript. All authors read, edited and approved the final manuscript.
